# Eyelid Molluscum Contagiosum Presenting as a Giant Nodule With Chronic Refractory Conjunctivitis

**DOI:** 10.7759/cureus.57018

**Published:** 2024-03-27

**Authors:** Suwarna Suman, Arushi Kumar

**Affiliations:** 1 Ophthalmology, All India Institute of Medical Sciences, Jodhpur, Jodhpur, IND; 2 Ear, Nose and Throat, Nalanda Medical College and Hospital, Patna, IND

**Keywords:** umblicated lesion, pox virus, follicular conjunctivitis, eyelid, molluscum contagiosum

## Abstract

Molluscum contagiosum is a benign cutaneous viral infection caused by a poxvirus, commonly seen in children and adolescents. It typically produces benign, self-limiting eruptions on the skin and mucous membranes, usually on the face, trunks, limbs, and genital areas. The eyelid is the most common site of ocular lesions, less commonly conjunctiva.Eyelid Lesions are typically small papules (two to six mm) with central depressions, or maybe non-umbilicated. Patients with immunodeficiency may have an atypical giant lesion or widely disseminated lesions. We present a case of eyelid molluscum contagiosum presenting with an unusually large nodule with two depressions associated with chronic follicular conjunctivitis in a three-year-old otherwise healthy child. Eyelid lesions were removed surgically. The conjunctival follicular reaction was completely resolved after one month of surgical excision. A histopathological examination confirmed the diagnosis.

## Introduction

Molluscum contagiosum (MC) is a viral infection of skin and mucous membranes caused by a poxvirus, a DNA virus replicating in the cytoplasm of epidermal cells [1]. It typically produces benign, self-limiting eruptions on the skin and mucous membranes, commonly seen on the face, trunks, limbs, and genital areas. It usually affects children and adolescents, and adults with immunodeficiency [2]. The eyelid is the most common site of ocular lesions, less commonly conjunctiva [3]. Eyelid lesions are typically small papules (two to six mm) with central depressions or may be non-umbilicated [4]. Patients with primary immunodeficiency, HIV infection, or patients on immunosuppressant therapy may have an atypical giant lesion or widely disseminated lesions [5-8]. Here, we present a case of molluscum contagiosum of the eyelid in a three-year-old otherwise healthy child presenting with an unusually large nodule with two depressions associated with chronic follicular conjunctivitis not responding to treatment.

## Case presentation

A three-year-old girl child presented with a three-week history of painless mass, gradually increasing in size on her left upper eyelid. There was a history of redness, watering, and discomfort in the same eye for two months, for which she was advised topical antibiotics, anti-allergic, and artificial tear eye drops by several local practitioners but no improvement was noticed. The child’s past medical and family history was unremarkable. On examination, two pitted nodular lesions were detected on the left upper eyelid near the lid margin (Figure 1A). The larger one was about 10 mm x 8 mm x 6 mm in size, umbilicated, non-tender, and mobile; the other was smaller about 3 mm x 2 mm x 2 mm in size. The conjunctiva was hyperaemic with intense follicular reaction in the lower fornix (Figure 1B). The rest of the anterior segment examination was within normal limits. No similar lesions were present on other parts of the patient’s body. A diagnosis of left eye molluscum contagiosum with unilateral follicular conjunctivitis was made and advised for excisional biopsy. Both the papules were excised. Beneath the larger nodule, one more papule was present in the substance of the lid; was removed completely (Figure 1C). Histopathological examination revealed numerous inclusion bodies. At postoperative 15-day follow-up, the conjunctival follicular reaction was reduced and completely regressed after one month (Figure 1D). On 12 months follow-up no recurrence was observed.

**Figure 1:** Clinical photographs (A) A large nodular lesion with two depressions and a small papule in the upper eyelid. (B) Follicular reaction in the lower fornix. (C) Three excised papules. (D) Postoperative image showing regression of conjunctival follicular reaction.

## Discussion

The eyelid is the most common site of ocular molluscum contagiosum, less commonly conjunctiva, and rarely cornea [3]. Eyelid lesions are typically yellowish pink, raised, small papules (2-6 mm) with central depressions; or maybe non-umbilicated [4]. The diagnosis of eyelid lesions is usually clinical based on characteristic features of MC, however, it is difficult in cases with atypical presentation. Eyelid lesions are variable; they may not show umbilication and tend to be larger and flatter, especially located away from the eyelid margins, resembling a sebaceous cyst [4]. Giant or atypical lesions are reported in patients with AIDS or patients using immunosuppressive therapy [4,8]. In this case, the patient presented with a giant nodule located at the lid margin and showed double umbilication in an otherwise healthy child. A solitary large lid lesion should be differentiated from basal cell carcinoma, papilloma, chalazion, keratoacanthoma, blepharitis, and wart. Secondary infection or ulceration in the lesions may further complicate the diagnosis and may need histopathological confirmation [9,10].

Eyelid lesions may be associated with chronic follicular conjunctivitis or keratoconjunctivitis and are believed to be due to toxicity or hypersensitivity reaction to the viral proteins shed from the lid lesion into the tear film [10]. Corneal involvement occurs as punctate keratopathy or subepithelial infiltrates and corneal pannus in long-standing cases [4,6].

Molluscum contagiosum is an easily overlooked cause of chronic unilateral conjunctivitis refractory to routine treatment [4]. The initial inconspicuous or atypical eyelid lesions may be the cause of delay in diagnosis and treatment that might facilitate the spread of infection and scarring. In this case, there was also a long history of chronic conjunctivitis not responding to treatment before the parents noticed the nodule. Charteris et al., in a retrospective analysis of 35 patients with molluscum contagiosum, found that only 60% of the patients were diagnosed at the time of initial presentation, and delay in diagnosis of ocular MC was statistically significantly higher among patients with conjunctivitis in comparison to the non-conjunctivitis patients [5]. A careful examination of the eyelid margin is essential in patients with unilateral chronic follicular conjunctivitis, as a small inconspicuous lesion may be hidden behind the lashes.

Excision of the eyelid lesions is the preferred treatment option as it prevents recurrence and scaring [11]. Other treatment options are curettage, cryotherapy, and cautery. Surgical removal results in the resolution of anterior segment inflammation. Topical chemical agents like salicylic acid, Silver nitrate, and potassium hydroxide solution have been shown to be effective in cutaneous lesions [12]. Topical antiviral agent cidofovir (5%) or intralesional and systemic interferon-alpha has been used to treat resistant cases in immunocompromised patients [13].

## Conclusions

In summary, the patient described herein had an atypical presentation of eyelid molluscum contagiosum. The patient presented with an unusually large nodule with two depressions associated with chronic follicular conjunctivitis. The atypical appearance of the lesion and a variable ocular involvement may complicate the diagnosis. A careful examination of the eyelid and early recognition of the lesion is essential to prevent delay in diagnosis and treatment. Eyelid lesions were removed surgically in this case.

## References

[1] Meza-Romero R, Navarrete-Dechent C, Downey C (2019). Molluscum contagiosum: an update and review of new perspectives in etiology, diagnosis, and treatment. Clin Cosmet Investig Dermatol.

[2] Serin Ş, Bozkurt Oflaz A, Karabağlı P, Gedik Ş, Bozkurt B (2017). Eyelid Molluscum Contagiosum Lesions in Two Patients with Unilateral Chronic Conjunctivitis. Turk J Ophthalmol.

[3] Schornack MM, Siemsen DW, Bradley EA, Salomao DR, Lee HB (2006). Ocular manifestations of molluscum contagiosum. Clin Exp Optom.

[4] Curtin BJ, Theodore FH (1955). Ocular molluscum contagiosum. Am J Ophthalmol.

[5] Charteris DG, Bonshek RE, Tullo AB (2005). Ophthalmic molluscum contagiosum: clinical and immunopathological features. Br J Ophthalmol. 1995;79: 476-481.Espinoza GM and Lueder GT. Conjunctival pyogenic granulomas after strabismus surgery. Ophthalmology.

[6] Ritterband DC, Friedberg DN: Virus infections of the eye (1998). Virus infections of the eye. Rev Med Virol.

[7] Kurwa HA, Marks R (1995). Protracted cutaneous disorders in association with low CD4+ lymphocyte counts. Br J Dermatol.

[8] Hicks CB, Myers SA, Giner J (1997). Resolution of intractable molluscum contagiosum in a human immunodeficiency virus-infected patient after institution of antiretroviral therapy with ritonavir. Clin Infect Dis.

[9] Örnek K, Onaran Z, Koçak M (2014). Giant eyelid molluscum contagiosum presenting as preseptal cellulitis. J Paediatr Child Health.

[10] Alrajeh M, Alessa D, Maktabi AM, Al Alsheikh O (2018). Eyelid molluscum contagiosum presenting as a giant solitary ulcerating mass. Saudi J Ophthalmol.

[11] Osadebe LU, Li Y, Damon IK, Reynolds MG, Muyombwe A, Gappy C (2014). Ocular molluscum contagiosum atypical clinical presentation. Pediatr Infect Dis J.

[12] Scheinfeld N (2007). Treatment of molluscum contagiosum: a brief review and discussion of a case successfully treated with adapelene. Dermatology Online J.

[13] Hourihane J, Hodges E, Smith J, Keefe M, Jones A, Connett G (1999). Interferon alpha treatment of molluscum contagiosum in immunodeficiency. Arch Dis Child.

